The article "Research on the spatial temporary evolution of urban expansion in Xining city and its surrounding areas based on Landsat time series data" was published in 2024. Journal: Heliyon.

# Research on the spatial temporary evolution of urban expansion in Xining city and its surrounding areas based on Landsat time series data^☆^

**DOI:** 10.1016/j.heliyon.2024.e24846

**Published:** 2024-01-17

**Authors:** Xiaomin Cao, Xiaohong Gao, Runxiang Li

**Affiliations:** a Qinghai Meteorological Observatory, Xining, 810001, China; b College of Geographical Sciences, Qinghai Normal University, Xining, 810008, China; c Key Laboratory of Tibetan Plateau Land Surface Processes and Ecological Conservation (Ministry of Education), Qinghai Normal University, Xining, 810008, China; d Qinghai Provincial Key Laboratory of Physical Geography and Environmental Process, College of Geographical Science, Qinghai Normal University, Xining, 810008, China

**Keywords:** Random forest, Landsat series images, Spatio temporary consistency check, Land use transfer matrix, Nuclear density, Xining city and surrounding areas

## Abstract

Quantitative analysis of the process of urban expansion and evolution is of great practical significance for the future planning and development potential of valley cities. Based on GEE cloud platform and Landsat satellite data, this paper analyzed the spatio-temporal change characteristics and transfer rules of land cover in Xining City and its surrounding areas in the past 33 years by using random forest algorithm, spatio-temporal consistency test, land use dynamic attitude, transfer matrix and transfer hot spot analysis methods. The results show that the accuracy range of the preliminary classification of construction land is improved by 1.57%–3.53 % by using the spatio-temporal consistency test algorithm. The characteristics of land cover change in the study area are mainly the increase of construction land and forest area, the decrease of cultivated land and grassland area, the small change of water body and unused land, and the change of land cover type from cultivated land to urban construction land is prominent. The hot areas of construction land have gradually shifted from the central and eastern districts of the city in 1987 to the hot areas dominated by the Haihu New District of the West of the city, the Biological Park and the higher education base of the North District of the city, the South New District of the city, Duoba Town and the Ganhe Industrial Park in 2019.

## 1 Introduction

A city is the political, economic, and cultural core of a region. Urban space provides the most basic venue for related socio-economic activities and serves as a landmark for its socio-economic development, fully demonstrating the current status and level of development of the region and its country [1]. With the increase of urban population, the acceleration of urbanization process, the increasing consumption level of urban population, and the demand for high-quality living conditions, the urban spatial pattern has undergone significant evolution over time, ultimately leading to an increase in the density of building land within the city. Industrial and low-density residential land in the old city has been developed into high-density residential and commercial land, The agricultural land around the urban area is constantly being occupied and transformed into urban construction land. Studying the size of urban land use, growth trends, and proportion of the total research area can evaluate the suitability of urban development and changes, as well as the degree of harmonious coexistence between humans and nature. It is of great significance for exploring current urban development issues and future urban development planning and construction [2,3]. Accurately grasping the historical evolution of urban land cover plays a crucial role in enhancing urban competitiveness and sustainable development in the future [4,5].

The article "Research on the spatial temporary evolution of urban expansion in Xining city and its surrounding areas based on Landsat time series data" was published in 2024. Journal: Heliyon.

Li et al. [6] studied the changes in urban expansion in Beijing over the past 30 years based on long-term Landsat data from 1984 to 2013. During this process, the random forest algorithm was used to classify remote sensing images from year to year, obtaining annual data on urban development, and conducting time consistency tests to improve classification accuracy.Yang et al. [3] used Shenzhen as the research area and selected 18 Landsat 3/5/7/8 images from 9 issues from 1979 to 2020 as the main data source to extract the proportion of impermeable surfaces as reference data. They combined the average center of impermeable surfaces, standard deviation ellipse, and landscape pattern index to analyze the spatio-temporal distribution pattern of impermeable surfaces in Shenzhen. Xia et al. [7] used Landsat series remote sensing images as the data source to extract urban construction land. Combining urban expansion evaluation indicators and socio-economic statistical data, they analyzed the spatio-temporal characteristics and driving factors of urban expansion in Hefei in the past 20 years. Zhao et al. [8] used artificial visual interpretation combined with Google historical image correction to extract built-up areas based on remote sensing images of Taiyuan City from 1973 to 2020. They introduced indicators such as compactness, expansion intensity, expansion speed, and center of gravity migration model to analyze the spatio-temporal evolution characteristics of the built-up areas in Taiyuan City over the past 50 years. Most of the above studies only used multi period Landsat data rather than long-term time series data to analyze the spatio-temporal pattern of urban expansion, which makes it difficult to reflect the dynamic process of urban expansion at a high time frequency.

The article "Research on the spatial temporary evolution of urban expansion in Xining city and its surrounding areas based on Landsat time series data" was published in 2024. Journal: Heliyon.

This study takes the urban area of Xining and its surrounding areas as the research area. With the support of the GEE cloud platform, based on the Landsat satellite long time series image data from 1987 to 2019 for the past 33 years, using random forest algorithm, feature parameter optimization, and spatio-temporal consistency testing methods, we plan to obtain a land cover dataset for the research area for 33 years; On this basis, land use dynamics, transfer matrix, and transfer hotspot analysis methods will be used to quantitatively study the spatio-temporal changes and transfer laws of land cover in Xining City and surrounding areas from 1987 to 2019, explore the urban evolution process, and provide data support and decision-making basis for the future sustainable development of urban green in the research area.

## 2 Research area and data source

### 2.1 Overview of the research area

The administrative scope of Xining City covers five districts and two counties, namely Chengdong, Chengzhong, Chengxi, Chengbei, Huangzhong Huangyuan and Datong, with a total area of 7660 km^2^. Xining urban area is located in Huangshui, Beichuan, Nanchuan and belongs to a narrow east-west valley type city. Huangshui passes through the city from west to east, and the Beichuan River and Nanchuan River respectively converge into Huangshui from the north and south in the urban area. In order to facilitate the study of urban expansion, the scope of Xining City and its surrounding areas is defined as: extending a certain range outward based on the Xining urban area/built-up area, as the scope of this study. The geographical location of this study is 36°10′-36°50′N, 101°20′-102°10′E, with an area of 1636 km^2^ and an altitude of 2102–2848 m. Its scope includes four districts under the jurisdiction of Xining City, Huangzhong, Datong and Huangyuan. County.In addition, it also includes some areas of Huzhu County and Ping'an County. The Landsat image track number of the covered research area is 132/035, which is an entire scene image. The location of the research area is shown in Fig. 1. The built-up area of Xining urban area is located in the plain areas of the Huangshui River, Beichuan River and Nanchuan River valleys, surrounded by low mountains and hills. The overall terrain is characterized by high in the west and low in the east, and low between high and low in the north and south, with hills distributed on both sides of the Huangshui main stream, as well as on the east and west sides of the Beichuan River and Nanchuan River. The east-west and north-south directions are characterized by flat valley plains, which are suitable for urban construction.

The article "Research on the spatial temporary evolution of urban expansion in Xining city and its surrounding areas based on Landsat time series data" was published in 2024. Journal: Heliyon.

**Fig. 1:** Location of the study area.

### 2.2 Data source and preprocessing

Landsat TM/ETM plus/OLI (Land Resources Satellite Series) data, due to its global coverage, long period historical archive data, and high spatial resolution (30 m), enables it to monitor long-term land cover changes, becoming an important data source for urban expansion research.

The cloud cover of 377 Landsat images selected in this paper is all lower than 10 %, and this data has been processed into L1T products, as shown in Fig. 2. The SRTM DEM V3 (Shuttle Radar Topography Mission) data was collected from the SRTM system carried by the US space shuttle Endeavour, with a spatial resolution of 30 m. The dataset has been filled with depressions [9]. NPP-VIIRS is non radiometric night stable light data released by the National Geographic Data Center of the United States [10]. FLDAS (Famine Early Warning Systems Network Land Data Association System) is a land data assimilation system established to assist developing countries with sparse data in training data. It includes information on many climate related variables, such as soil moisture, atmospheric humidity, evapotranspiration, total precipitation rate, etc. [11]. All the above data are directly called from the GEE cloud platform. In addition, NDVI (plant flourishing period and withering period), NDBI, EVI, NDWI, slope, aspect, and texture information are calculated separately to improve the classification accuracy of vegetation and construction land.

**Fig. 2:** Temporary distribution of Landsat images used in this study (Cao et al., 2020).

## 3 Research methods

### 3.1 Random forest classification method

According to the National Remote Sensing Monitoring Land Use/Cover Classification System and combined with the distribution characteristics of land use and land cover in the study area, the land cover classification system of the study area was determined into six categories: cultivated land, forest land, grassland, water area, urban and rural industrial and mining residential construction land and unused land.

The Random Forest (RF) algorithm was proposed by Breiman (2001) [12]. It is a classification model based on the CART (Classification and Regression Tree) decision tree and belongs to a new type of machine learning algorithm [13]. The basic principle is a decision tree model based on the Bagging ensemble learning framework, which covers many trees, each of which provides important classification results. The generation rules for each tree are as follows: (1) If the training set size is *N*, for each tree, *N* training samples are randomly and selectively selected from the K training set, which is used as the training set for the tree. Repeat *K* times to generate a group of training sample sets. (2) If the sample dimension of each feature is *M*, specify a constant *m ≤ M*, and randomly select *m* features from the *M* features. (3) Utilize *m* features to maximize the growth of each tree without pruning.

The article "Research on the spatial temporary evolution of urban expansion in Xining city and its surrounding areas based on Landsat time series data" was published in 2024. Journal: Heliyon.

Based on a random forest classifier, input a sample set and feature parameters to classify the land cover of the study area year by year. In this process, optimizing the distribution of sample space and optimizing feature parameters are two important steps to improve classification accuracy. In order to reflect the randomness and representativeness of sample spatial distribution, it is necessary to optimize it during the classification process. The selection of training and validation samples was previously determined based on the random number function, but this cannot ensure that the training and validation samples are uniformly distributed in space and maintain a consistent proportion for each class of samples. Therefore, in the GEE platform, the above problem is solved by setting a threshold while calling the random number function. Entering too many feature variables into the same model will result in data redundancy, so optimization is needed in model parameter tuning [14].The feature variables or feature parameters selected in this paper mainly include spectral features, spectral feature index, terrain features, texture features, climate factors and night light data, as shown in Table 1.

**Table 1:** Original features parameters and the optimized feature parameters.

Feature type	Original feature parameters	Optimized feature parameters
Spectral characteristics	Band1, Band2, Band3, Band4, Band5, Band6, Band7, Band8, Band9, Band10, Band11, Band12, EVI, RVI, NDBI, NDVI, NDWI, csNDWI	Band2, Band3, Band4, Band5, Band6, Band7, Band10, Band11, EVI, NDBI, NDVI, NDWI
Topographical features	DEM, slope, aspect, hillshade	DEM, aspect, slope
Texture features	Ent, maxcorr, asm, inertia, contrast, dent, idm, corr, var, dvar, savg, prom, imcorr, send, dis Shade	Best 1 type
Climatic factors	Evap_ Tavg, LWdown_ F_ Tavg, Lwnet_ Tavg, Psurf_ F_ Tavg Qair_ F_ Tavg, Qg_ Tavg, Qh_ Tavg, Qle_ Tavg, Qs_ Tavg Qsb_ Tavg, RadT_ Tavg, Rainf_ F_ Tavg, Wind_ F_ Tavg, SoilMoi00_ 10 cm_ Tavg, SoilMoi10_ 40 cm_ Tavg SoilMoi100_ 200 cm_ Tavg, SoilMoi40_ 100 cm_ Tavg, SoilTemp00_ 10 cm_ Tavg, SoilTemp10_ 40 cm_ Tavg, SoilTemp100_ 200 cm_ Tavg, SoilTemp40_ 100 cm_ Tavg, SWdown_ F_ Tavg, Swnet_ Tavg, Tair_ F_ Tavg	Best 1 type
Lighting data	NPP-VIIRS	NPP-VIIRS

The article "Research on the spatial temporary evolution of urban expansion in Xining city and its surrounding areas based on Landsat time series data" was published in 2024. Journal: Heliyon.

### 3.2 Classification post-processing and spatiotemporal consistency testing

After using the random forest method to classify annual Landsat images, a preliminary land cover classification map of the study area was obtained for a long time series (33 years). However, in these preliminary classification results, the salt and pepper phenomenon caused by the same object but different spectra of the images was severe, especially in the Landsat images of earlier years before 2000, where the quality was poor and the debris patch phenomenon was more severe, which required post-classification processing. In addition, for long time series data, spatiotemporal consistency testing, namely temporal consistency testing and spatial consistency testing, is also required. Time consistency testing refers to checking for errors in patch attributes generated by land cover types during the classification process in long-term time series classification research. Space consistency testing refers to the inference process for correct patch attribute types during the time consistency testing process [14].

To this end, the Majority Filter of ArcGIS software is first used to classify and process the annual classification results to eliminate debris patterns. On this basis, spatio-temporal consistency testing is conducted. Due to the involvement of six major types of land cover in the study area, during the 33 year spatio-temporal change process, complex mutual transformations occurred between different types of land cover, making it impossible to test the spatiotemporal consistency of each type of land cover. Therefore, in this study, only spatio-temporal consistency testing was conducted on urban and rural residential construction land, aiming to test whether the annual changes in the long-term series obtained conform to the objective laws of urban development, Its core is to distinguish true changes and classification errors from long-term time series information, improve the initial classification results of urban and rural residential construction land, and obtain more reliable time series classification data.

This study drew inspiration from the time consistency testing method proposed by Li et al. [6] and made localized modifications. The algorithm is implemented using Matlab 2017 software. The spatio-temporal consistency test includes temporal filtering and logical reasoning. The specific reasoning process is shown in Fig. 3.

(1) Time filtering: The main purpose of implementing time filtering is to filter out noise or classification errors introduced by single period images in the time series.

**Fig. 3:** Schematic diagram of temporary and spatial consistency test for unban land.

The article "Research on the spatial temporary evolution of urban expansion in Xining city and its surrounding areas based on Landsat time series data" was published in 2024. Journal: Heliyon.

In the above time filtering, the main problem is to solve the problem of classification consistency, and the key to implementation is the time domain window and probability judgment on the time series. Therefore, based on the probability function proposed by Li et al. [6], see formula (1).

(1) $$prob_{i}=\frac{\sum_{j=i-T_{w}}^{j=i+T_{w}}con\left(L_{j}=L_{i}\right)}{1+2\times T_{w}}$$

In the formula: $prob_{i}$ represents the probability function, represents the i pixel, represents the $T_{w}$ time domain window, $L_{j}L_{i}$ represents the target year, represents the neighborhood year, and con() represents the judgment function. The conversion rule for current category label discrimination: when $L_{j}$ = $L_{i}$, the con() return value is 1, otherwise it is 0; And set the threshold to 0.5. When it is $prob_{i}$ greater than 0.5, no category correction will be performed; When it is $prob_{i}$ less than 0.5, perform category correction.

(2) Logical reasoning: After the process of time filtering, some misclassified pixels can be corrected, but there are still logical irrationality situations in the long time series. That is, if the alternating years of construction land and non construction land occur, it is considered unreasonable. Therefore, it is necessary to logically rationalize them in the time series.

The accuracy evaluation uses confusion matrix, also known as error matrix, to calculate relevant indicators based on it. Specifically, these accuracy indicators include overall classification accuracy (OA), Kappa coefficient, mapping accuracy (PA), and user accuracy (UA), which reflect the accuracy of land cover classification from different perspectives [15,16].

### 3.3 Analysis of land use dynamics and transfer matrix

Based on dynamic degree indicators, it is possible to quantitatively study the specific changes in a certain type of land cover area in a certain region in relevant time dimensions. It can be called a dynamic index of a certain type, and has great value in studying the specific speed of land cover change and predicting subsequent change trends [17]. The expression is shown in formula (2):

(2) $$K=\frac{U_{b}-U_{a}}{U_{a}}\times \frac{1}{T}\times 100\%$$

In the formula: K is the annual change rate of the type in the analysis area; $U_{a}$ To analyze the data of a certain type of land cover area in the initial period of the region; Data $U_{b}$ on the coverage area of a certain type of land in the late stage; T For the purpose of research duration, years are generally used as the basic unit.

The transfer matrix refers to the area of objective things that transfer from one state to another. By quantitatively describing the transfer between various states, a land cover transfer matrix is formed, which intuitively reflects the transfer area and direction between different cover types, in order to reveal the changes in different land types [18,19]. The matrix expression can be found in formulas (3) and (4):

(3) $$S_{\left(t+1\right)}=P_{ij}\times S_{t}$$

In the formula: $S_{t}$ represents the $S_{\left(t+1\right)}$ land use status of the t-th period, and represents the land use status of the subsequent period of the t-th period; The mathematical expression for the transfer probability of $P_{ij}$ land use type i converted to type j in the subsequent period in the t-th period is generally [20]:

(4) $$P_{ij}=\left[\begin{array}{ccccc} p_{11} & p_{12} & p_{13} & \ldots \ldots & p_{1n}\\ p_{21} & p_{22} & p_{23} & \ldots \ldots & p_{2n}\\ p_{31} & p_{32} & p_{33} & \ldots \ldots & p_{3n}\\ \vdots & \vdots & \vdots & \vdots & \vdots \\ p_{n1} & p_{n2} & p_{n3} & \ldots \ldots & p_{nn} \end{array}\right]$$

Among them i,j=1,2,3⋯⋯,n, n is the number of types of land cover and meets two conditions: (1) $0\leq S_{ij}\leq 1$; (2) $\sum_{i}^{n}P_{ij}=1\left(i,j=1,2,3,\cdots ,n\right)$.

The article "Research on the spatial temporary evolution of urban expansion in Xining city and its surrounding areas based on Landsat time series data" was published in 2024. Journal: Heliyon.

### 3.4 Transfer hotspot analysis

In order to better analyze the spatial transfer characteristics of urban construction land, this article uses spatial point aggregation analysis, also known as hotspot analysis, to reflect its changes. The kernel density estimation method is often used for transfer hotspot analysis, which is easy to implement and can better reflect the distance attenuation effect in the spatial distribution of geographical phenomena. It conforms to the first law of geography and is the most commonly used hotspot analysis method [21]. The analysis of transfer hotspots consists of three aspects: transfer ratio, kernel density, and standard deviation ellipse.

Transfer ratio refers to the degree of conversion between other types of land and urban and rural residential construction land in each grid or grid unit, as calculated by formula (5).

(5) $$D=\frac{A_{u}-A_{e}}{A}\times 100\%$$

In the formula: D represents the transfer ratio to be calculated.The $A_{u}$ conversion of other land cover types representing the grid to the corresponding area of urban and rural residential construction land in the grid.The area $A_{e}$ representing the transformation of urban and rural residential construction land into other types of cover in the grid. A Represents the corresponding grid area.

The kernel density estimation method takes each sample point i (x, y) as the center, and calculates the density contribution value of each grid unit center point within the specified radius range (circle with bandwidth h as the radius) through the kernel function. The closer the grid unit center point within the search radius range is to the sample point, the greater its density contribution value [22]. The nuclear density can be used to analyze the hot spots where the density of construction land shifts [23]. The calculation is shown in formula (6).

(6) $$F_{n}\left(x\right)=\frac{1}{nh}\sum_{i=1}^{n}k\left(\frac{x-x_{i}}{h}\right)$$

In the formula: $F_{n}\left(x\right)$ represents the nuclear density value of the research area. $\left(x-x_{i}\right)$ Represents the distance $x_{i}$ between the estimated target grid center x and the bandwidth range grid sample points. H is used to describe the actual bandwidth. N is used to represent the number of samples in the bandwidth.

The article "Research on the spatial temporary evolution of urban expansion in Xining city and its surrounding areas based on Landsat time series data" was published in 2024. Journal: Heliyon.

The transfer hotspots show significant spatial differentiation in different periods, and standard deviation ellipses are used for spatial dynamic change analysis to observe the direction changes of land transfer [24]. Calculation can be found in (7), (8), (9), (10).

(7) $$\mu =\frac{\sum_{i=1}^{n}x_{i}}{n}\;v=\frac{\sum_{i=1}^{n}y_{i}}{n}$$

(8) $$\tan\;\theta =\frac{\left(\sum_{i=1}^{n}{x^{\prime }}_{i}^{2}-\sum_{i=1}^{n}{y^{\prime }}_{i}^{2}\right)+\sqrt{{\left(\sum_{i=1}^{n}{x^{\prime }}_{i}^{2}-\sum_{i=1}^{n}{y^{\prime }}_{i}^{2}\right)}^{2}+4{\left(\sum_{i=1}^{n}{x^{\prime }}_{i}^{2}{y^{\prime }}_{i}^{2}\right)}^{2}}}{2\sum_{i=1}^{n}x_{i}^{\prime }y_{i}^{\prime }}$$

(9) $$\delta_{x}=\sqrt{\frac{\sum_{i=1}^{n}{\left(x_{i}^{\prime }\;\cos\;\theta -y_{i}^{\prime }\;\sin\;\theta \right)}^{2}}{n}}$$

(10) $$\delta_{y}=\sqrt{\frac{\sum_{i=1}^{n}{\left(x_{i}^{\prime }\;\cos\;\theta -y_{i}^{\prime }\;\sin\;\theta \right)}^{2}}{n}}$$

μ and v respectively represent the average x and y coordinates of all points in the sample set, that is, the center of the ellipse, $x_{i}^{\prime }$ and $y_{i}^{\prime }$ are the relative coordinates of each sample point and the center of gravity. θ stands for the actual rotation Angle of the ellipse. The specific corner of the point distribution pattern can be obtained by combining tanθ. $\delta_{x}$ and $\delta_{y}$ represent the experimental standard deviation along the x axis and the experimental standard deviation along the y axis respectively [25].

Based on the Spatial Analyst Tools and Spatial Statistics Tools of ArcGIS 10.8, the transfer ratio, kernel density and standard deviation ellipse were calculated. On this basis, the hot spots of the transfer were further determined and analyzed.

## 4 Results and analysis

### 4.1 Accuracy evaluation result

Fig. 4 shows the accuracy evaluation results for four different scenarios from 1987 to 2019, with the blue area showing the overall classification accuracy of land cover using only spectral bands and spectral and topographic feature parameters, such as NDVI, RVI, NDWI, NDBI, EVI, DEM, Slope, and Aspect, year by year; The green line is the overall classification accuracy of land cover obtained year by year through four steps: optimizing the spatial distribution of samples, optimizing texture features and optimal windows, optimizing climate factors, and sorting feature parameters; The black line is the annual evaluation result of land cover classification accuracy after spatio-temporal consistency testing. It can be seen that after conducting spatio-temporal consistency testing on classified data, the overall accuracy of most years' data can be significantly improved, with an accuracy range of 1.57 %–3.53 % [14].

The article "Research on the spatial temporary evolution of urban expansion in Xining city and its surrounding areas based on Landsat time series data" was published in 2024. Journal: Heliyon.

**Fig. 4:** The results of Accuracy assessment.

### 4.2 Analysis of spatio-temporal changes in land cover in xining city and surrounding areas from 1987 to 2019

In order to deeply explore the characteristics of land cover changes in different time periods in the research area, based on the 33 year year by year land cover data obtained, urban and rural residential construction land was extracted and the area changes in adjacent years were analyzed. It was found that the three time nodes of 1993, 2003, and 2013 were the mutation years of urban and rural residential construction land changes [14]. Therefore, the period from 1987 to 2019 was divided into four time periods, namely 1987 to 1993 From 1993 to 2003, from 2003 to 2013, and from 2013 to 2019, dynamic changes in land cover were analyzed.

Using the statistical function of ArcGIS, the land cover classification grid data of the study area in 1987, 1993, 2003, 2013, and 2019 were used to calculate the land cover area of the corresponding years. Use Excel to calculate the proportion of each type of area, and according to formula (2), calculate the annual change rate of land cover in the study area from 1987 to 2019 and its four periods, as shown in Table 2 and Fig. 5.

**Table 2:** The area, property and annual rate of change of land cover types in the study area from 1987 to 2019.

Land cover type	1987		1993		2003		2013		2019	
	area (km^2^)	Proportion (%)	area (km^2^)	Proportion (%)	area (km^2^)	Proportion (%)	area (km^2^)	Proportion (%)	area (km^2^)	Proportion (%)
Cropland	686.74	41.97	297.27	18.16	447.16	27.32	494.22	30.21	369.08	22.55
Forest	138.75	8.48	471.60	28.82	402.98	24.62	314.18	19.20	293.91	17.96
Grassland	731.84	44.72	772.96	47.22	659.27	40.28	583.98	35.68	626.5	38.29
Water	17.33	1.06	17.47	1.07	7.29	0.45	8.41	0.51	7.11	0.43
Construction land	54.67	3.34	70.09	4.29	114.21	6.99	228.45	13.96	334.15	20.43
Bare land	7.09	0.43	7.03	0.44	5.51	0.34	7.18	0.44	5.75	0.34
total	1636.42	100.00	1636.42	100.00	1636.42	100.00	1636.42	100.00	1636.42	100.00

Land cover type	1987–1993		1993–2003		2003–2013		2013–2019		1987–2019	
	Area of variation (km^2^)	Land cover Annual change rate (%)	Area of variation (km^2^)	Land cover Annual change rate (%)	Change area (km^2^)	Land cover Annual change rate (%)	Area of variation (km^2^)	Land cover Annual change rate (%)	Area of variation (km^2^)	Land cover Annual change rate (%)
Cropland	−389.47	−9.45	149.9	5.04	47.06	1.06	−125.14	−4.22	−317.80	−1.44
Forest	332.85	39.96	−68.63	−1.46	−88.80	−2.20	−20.27	−1.07	155.17	3.49
Grassland	41.12	0.93	−113.70	−1.47	−75.29	−1.14	42.52	1.21	−105.41	−0.45
Water	0.14	0.13	−10.15	−5.81	1.12	1.47	−1.30	−2.56	−10.29	−1.84
Construction land	15.42	4.73	44.11	6.28	114.24	9.99	105.70	7.73	279.76	15.99
Bare land	−0.06	0.09	−1.53	−2.14	1.67	2.79	−1.51	−3.52	−1.43	−0.63

The article "Research on the spatial temporary evolution of urban expansion in Xining city and its surrounding areas based on Landsat time series data" was published in 2024. Journal: Heliyon.

**Fig. 5:** Area percentage of land cover types in the study area from 1987 to 2019.

From Tables 2 and it can be seen that the research area is mainly composed of cultivated land and grassland types. In 1987, the two types accounted for 41.97 % and 44.72 % of the total area, followed by forest land, accounting for 8.48 %. Urban and rural residential construction land, water bodies, and unused land accounted for 3.34 %, 1.06 %, and 0.43 %, respectively. In 2019, the proportion of grassland and arable land in the total area decreased to 38.29 % and 22.55 %, respectively, while the proportion of urban and rural residential construction land and forest land increased to 20.43 % and 17.96 %, respectively. There was little change in water bodies and unused land.

From 1987 to 2019, the area of cultivated land and grassland showed a decrease, with the largest decrease in cultivated land area, which was the largest change in area among all types. From 686.90 km^2^ in 1987 to 369.09 km^2^ in 2019, the area has decreased by 317.81 km^2^, and the annual change rate of land cover is −1.44 %. On the contrary, both construction land and forest land types show an increase in area, and the increase in construction land area is greater than that of forest land. From 1987 to 2019, the area of construction land increased from 54.67 km^2^ to 334.44 km^2^, with an increase of 279.771 km^2^. Its proportion increased from 3.34 % to 20.43 %, with an annual change rate of 15.99 %. The forest area increased by 155.1 km^2^, while the grassland area decreased by 105.4 km^2^, with annual change rates of 3.49 % and −0.45 %, respectively. The proportion of unused land and water bodies is relatively small and has remained basically unchanged for 33 years. The analysis shows that the construction land in the research area has experienced the largest changes from 1987 to 2019, followed by forest land and cultivated land.

The article "Research on the spatial temporary evolution of urban expansion in Xining city and its surrounding areas based on Landsat time series data" was published in 2024. Journal: Heliyon.

### 4.3 Transition matrix analysis

In order to more intuitively and deeply reflect the transfer direction of various land types in the study area at different periods, based on five land cover classification grid data from 1987, 1993, 2003, 2013, and 2019, the area of each land cover type in the five years was calculated. At the same time, the merging of forest and grassland, water bodies, and unused land were merged. Based on the transfer matrix formula (3), a program was written in Python language to implement the Sangji map, as shown in Fig. 6, Intuitively express the changes in the proportion of area of each type from 1987 to 2019 and the mutual conversion relationship between each type.

**Fig. 6:** Sankey diagram of the transition between different land cover types in the study area from 1987 to 2019 Note: CUL represents cultivated land, VEG represents grassland and forest land, BUL represents construction land, OTH represents water bodies and unused land.

From Fig. 6, it can be seen that the proportion of urban and rural residential construction land in Xining City and surrounding areas has been increasing from 1987 to 2019, but the main increase was from 2003 to 2019, especially in the nearly 7 years from 2013 to 2019. The increase was mainly from the conversion of arable land, with a small portion being from forest land. The loss of arable land is not simply converted into urban and rural residential construction land, but also mainly turns to forest and grassland land, with the most significant shift from 1987 to 1993. About 50 % (1/2) of the arable land column showed a shift to forest and grassland land, which is closely related to the local government's greening of the north and south mountains in Xining City during this period; Secondly, from 2013 to 2019, about 1/4 of them flowed to forest and grassland land, 1/4 to construction land, and 2/4 remained unchanged. Further analysis shows that there is a significant mutual transformation between cultivated land, forests, and grasslands from 1987 to 2019, manifested as a shift from cultivated land to forests and grasslands from 1987 to 1993 and from 2013 to 2019. From 1999 to 2003 and from 2013 to 2019, the shift from forests and grasslands to cultivated land was the main trend.

From the research results, it can be seen that the pilot project of returning farmland to forests was launched in 1999, and the project was fully launched in 2002. It has been 19 years since then. However, in the early stages of the project of returning farmland to forests (1999–2003), due to the lack of a coordinated plan for the comprehensive development of agriculture, forestry, and animal husbandry, rational allocation of land resources, and comprehensive development. There are some problems in the implementation of the plan for returning farmland to forests and grasslands, which has not been scientifically proven. The plan is only limited to the implementation of project funds, and the operability is not strong, and it has not been implemented according to the plan [26]. In order to consolidate the previous achievements, a new round of returning farmland to forests (2014–2020) was comprehensively launched in 2014.

The article "Research on the spatial temporary evolution of urban expansion in Xining city and its surrounding areas based on Landsat time series data" was published in 2024. Journal: Heliyon.

### 4.4 Spatial and temporal expansion of urban construction land in xining city and its surrounding areas in the past 33 years

Based on 33 years of annual data on the area of urban and rural residential construction land, a map algebra tool with spatial analysis function was used to draw a gradual expansion and change map of urban construction land in Xining City from 1987 to 2019, using the urban and rural residential construction land in 1987 as the reference year, as shown in Fig. 7. This figure shows the expansion process of urban construction land in Xining City over the past 33 years, and the gradient of the legend from yellow to blue represents the annual expansion process of construction land. The yellow area represents urban land from earlier years (1987 as the base year), while the blue area represents newly developed urban land. The urban development of Xining City in the past 33 years can be summarized as follows: (1) Controlled by the terrain pattern of the research area, it expands outward along the valley plain on both sides of the X shaped river skeleton on the basis of the original urban area. (2) The expansion of urban space is limited by the corresponding terrain and river valley trends, and the expansion process is to expand from the center of the original built-up area along the direction of Huangshui, Beichuan River, and Nanchuan River to the east west, north, and south directions respectively. (3) In addition to expanding along the Huangshui River, Beichuan River, and Nanchuan River, cities have also gradually expanded along the Kangchengchuan and Gangou River valleys on the south bank of Huangshui River, developing into Ganhe Industrial Park and Xizhuang, respectively. At the same time, it expands along the Shatang River on the north bank of Huangshui to Huzhu County.

**Fig. 7:** Urban expansion of the study area and its local area display (1987–2019).

From 1987 to 2019, the overall planning and development direction of Xining City gradually evolved from the initial eastward and southward development to westward and northward development. The city is expanding eastward and has connected to Xining Ping'an District. The city gradually expands westward to connect with Xining Huangzhong Duoba Town. The expansion of the city to the north and south has strengthened the development of Datong County, the southern part of Huangzhong County, and the Ganhe Park. The gradual development of the city to the east and northeast has also connected Xining City with Ping'an County and Huzhu County.

The article "Research on the spatial temporary evolution of urban expansion in Xining city and its surrounding areas based on Landsat time series data" was published in 2024. Journal: Heliyon.

### 4.5 Analysis of hot spots of urban transfer in xining city and its surrounding areas from 1987 to 2019

Based on the analysis method of transfer hotspots, the spatial analysis function of ArcGIS is used to create 1 km✕1 km grids based on the land cover data of the five phases mentioned above. Based on this 1 km grid unit, the transfer patterns of urban expansion centers in different periods are studied. Firstly, based on a 1 km grid, using map algebra and regional statistical tabulation in spatial analysis tools, combined with the transfer ratio formula (5), the transfer ratio is calculated and divided into 10 levels at equal intervals. The higher the level, the larger the absolute area of other land transferred to construction land, and vice versa, as shown in Table 3.

**Table 3:** Classification level of the transfer of other land type to construction land (%).

	grade									
	0	1	2	3	4	5	6	7	8	9
Transfer ratio	0	0∼8	8∼16	16∼24	24∼32	32∼40	40∼48	48∼56	56∼64	64∼72

Using ArcGIS software, the kernel density was calculated by using the transfer ratio column attribute, and the standard deviation ellipse was calculated by the direction distribution of the measured geographical distribution, so as to explore the hot areas where the urban expansion land transfer occurred.Fig. 8 shows the spatial distribution rules of the transfer of other land to urban construction land and the changes of transfer hotspots in four different time periods from 1987 to 2019. The specific performance is as follows:(1) Fig. 8a is from 1987 to 1993, the transfer of other land to construction land, with the central urban area and the Eastern urban area as the two main centers, and the transfer density of the eastern urban area is higher, while the western urban area has a small amount of land transfer, showing a point-like transfer pattern, the transfer level is between 2 and 3, and the development direction is east-west. (2)Fig. 8b is from 1993 to 2003, the transfer centers of other land to construction land in the whole research area expanded from 2 centers in the previous stage to 4 centers. The transfer density of the original urban center developed somewhat, while the eastern district weakened somewhat, while there were two obvious expansion centers in the northern and southern districts, and the development direction was still east-west. However, there is a trend of increasing development in the north-south direction. (3)Fig. 8c is from 2003 to 2013, the transfer area of other land to construction land increased significantly, and the transfer area was more concentrated in the western district, the Huangzhong County, the southern district, in addition to the northern district, mainly for the construction of Haihu New District, the southern New District, the Ganhe Industrial Park, and the biological park in the northern district. The transfer grade of the west and south of the city is 6–9, and the development direction is northeast-southwest. (4) Fig. 8d is from 2013 to 2019, the transfer density of other land to construction land has been very low in the eastern part of the city and the transfer level is almost the lowest. The western and southern parts of the city with high transfer density have significantly weakened compared with the previous period, and the transfer level has also decreased from the original 8–9 level to 7-2 level, but the transfer density in the northern part of the city has increased and the transfer level has risen to a higher level. In general, from 1987 to 2019, the urban expansion of Xining City mainly focused on the development and construction of the west, north and south of the city, while the development of the east of the city has weakened with the passage of time due to space constraints, and the development direction is north south east west, and the scope is larger.

The article "Research on the spatial temporary evolution of urban expansion in Xining city and its surrounding areas based on Landsat time series data" was published in 2024. Journal: Heliyon.

**Fig. 8:** Hot spots and distribution of spatial transfer of other land type transformed to construction land in the study area from 1987 to 2019.

## 5 Conclusion and prospect

This article is based on the GEE cloud computing platform and uses pixel stitching technology to obtain Landsat long time series data for research areas with cloud cover less than 15 % from 1987 to 2019. Random forest machine learning methods are used, combining spectral features, spectral indices, texture information, nighttime light data, and climate data to optimize sample distribution, texture features, and optimal windows The preliminary results of 33 year land cover classification in the study area were obtained through four steps of climate feature selection and optimal feature variable determination. Research has shown that the accuracy of sample selection and distribution optimization are very important factors in improving classification accuracy, while the use of texture features, climate features, etc. can improve classification accuracy to a certain extent, but is not a key factor in improving classification accuracy.

The article "Research on the spatial temporary evolution of urban expansion in Xining city and its surrounding areas based on Landsat time series data" was published in 2024. Journal: Heliyon.

Based on previous research and taking into account the terrain and geomorphological characteristics of the study area, a spatio-temporal consistency testing algorithm suitable for construction land in river valley cities was implemented. The preliminary classification results of construction land were corrected through time consistency testing and logical reasoning algorithms. The final land cover data of Xining City and surrounding areas from 1987 to 2019 for 33 years were obtained and their accuracy was evaluated, The overall classification accuracy of the final classification data is 83.33 %∼94.03 %, and its accuracy range has been improved by 1.57 %∼3.53 %. Conducting spatio-temporal consistency testing on long-term continuous construction land classification data can effectively improve classification accuracy to a certain extent.

The evolution process of urban spatial expansion spatio-temporal pattern from 1987 to 2019 is manifested as follows: the built-up area consisting of the X shaped water system composed of Huangshui and Nanbei River as the skeleton gradually spreads and expands outward along both sides of the river valley, the urban land expansion in the two river valleys of Ganhegou and Kangchengchuan, the tributaries of Huangshui in the southwest direction, the expansion along the Shatangchuan River to the north of Huzhu, and the increase of rural residential land scattered on both sides of the river valley. The characteristics of land cover change are mainly manifested as an increase in the area of construction land and forest land, a decrease in the area of arable land and grassland, and a relatively small change in the area of water bodies and unused land. The analysis of transfer hotspots shows that from 1987 to 2019, the urban construction area of the research area gradually shifted from being a hot area in the middle and east of the city to a hot area mainly consisting of the Haihu New Area in the west of the city, the North of the city Biological Park and Higher Education Base, the South of the city New Area, Duoba Town, and the Ganhe Industrial Park. During this process, cultivated land gradually loses and transforms into urban construction land. However, there are still some shortcomings in practical applications. In the future, in-depth research is needed on the correlation between urban construction land and other ecological environments.

## Additional information

No additional information is available for this paper.

## CRediT authorship contribution statement

**Xiaohong Gao:** Software, Data curation. **Gao Xiaohong:** Methodology, Conceptualization. **Runxiang Li:** Validation.

The article "Research on the spatial temporary evolution of urban expansion in Xining city and its surrounding areas based on Landsat time series data" was published in 2024. Journal: Heliyon.

## Declaration of competing interest

The authors declare the following financial interests/personal relationships which may be considered as potential competing interests:Xiaomin Cao reports was provided by Qinghai Normal University. Xiaomin Cao reports a relationship with xiaomin Cao that includes: consulting or advisory, employment, funding grants, and paid expert testimony. If there are other authors, they declare that they have no known competing financial interests or personal relationships that could have appeared to influence the work reported in this paper.
